# A case report of pancreaticoduodenectomy with en bloc celiac axis resection

**DOI:** 10.1097/MD.0000000000042233

**Published:** 2025-07-25

**Authors:** Mengna Zhang, Bin Zhang, Ying’an Zhao, Anle Wu, Jiyun Zhu, Xuanlei Ren, Jianbo Zheng, Siming Zheng

**Affiliations:** a The First Affiliated Hospital, Zhejiang University School of Medicine, Zhejiang University, Hangzhou, Zhejiang Province, China; b Department of Hepatobiliary and Pancreatic Surgery, The First Affiliated Hospital of Ningbo University, Ningbo, Zhejiang Province, China; c Invasive Technology Department, The First Affiliated Hospital of Ningbo University, Ningbo, Zhejiang Province, China.

**Keywords:** hepatic artery embolization, neoadjuvant chemotherapy, pancreatic cancer, total pancreaticoduodenectomy, with combined arterial resection

## Abstract

**Objective:**

To summarize the clinical experience of a case report of pancreaticoduodenectomy (PD) with en bloc celiac axis (CA) resection for locally advanced pancreatic cancer.

**Methods:**

We retrospectively analyzed the clinical data of a patient with locally advanced pancreatic cancer who underwent PD with en bloc CA resection after neoadjuvant chemotherapy and embolization of the proper hepatic artery at the Department of Hepatopancreatobiliary Surgery of the First Affiliated Hospital of Ningbo University in May 2023. This study was approved by the ethics committee of the Ningbo First Hospital.

**Results:**

This case was operated on smoothly with an operative time of 535 minutes and intraoperative bleeding of approximately 800 mL. Only short-term elevation of hepatic aminotransferase appeared in the postoperative period, which was improved by hepatoprotective and symptomatic treatments. The patient was discharged from the hospital 20 days postoperatively, and no tumor recurrence occurred in the follow-up period.

**Conclusion:**

In patients with locally advanced pancreatic cancer with simultaneous invasion of the celiac trunk, common hepatic artery, and hepatic innominate artery, total PD with en bloc CA resection is safe and feasible in cases where neoadjuvant chemotherapy is effective and after establishing hepatic collateral circulation by preoperative embolization of the hepatic innominate artery. Meanwhile, more cases from more centers are needed to validate this conclusion.

## 1. Introduction

The incidence of pancreatic tumors has increased worldwide in recent years. American Cancer Society 2021 statistics show that pancreatic cancer ranks fourth in cancer-related mortality and sixth in China, and its cancer-related mortality is expected to continue to climb in 2030, an outcome that is closely related to the inability of most patients to undergo radical resection.^[1]^

The pancreas is anatomically deep and adjacent to large blood vessels in the upper abdomen. Pancreatic cancer starts insidiously but progresses rapidly with atypical symptoms. Therefore, when pancreatic cancer is diagnosed, it often has already invaded blood vessels, and most of the patients lose the opportunity of radical treatment by surgery.^[2]^ With the progress of drug treatment for pancreatic cancer, the development and application of imaging, pathological disciplines, and new surgical concepts, new opportunities, and advances have been brought to the treatment of pancreatic cancer, prompting surgeons to constantly challenge and break through the “forbidden zone” of pancreatic surgery. Radical pancreatic cancer surgery with combined venous resection has become an international consensus,^[3]^ but can radical pancreatic cancer surgery with combined arterial resection really benefit patients with locally advanced disease? This study has been extensively explored and validated. A case of total pancreaticoduodenectomy (PD) with combined arterial resection was recently performed at our center and is reported here for further discussion.

## 2. Case presentation

A 54-year-old female patient presented with vague pain in the middle and upper abdomen for more than 1 month without any obvious trigger or other discomfort. Examination showed “fasting blood glucose 17.46 mmol/L; serum CA199 44.3U/mL.” Abdominal ultrasound, MRI-enhanced pancreas, and CT-enhanced epigastric abdomen all showed head and neck pancreatic occupations of approximately 27 × 20 mm, suggesting a high probability of pancreatic cancer, which involves the portal vein (PV), celiac trunk, and its branches. The tail of the pancreatic body was atrophied, the main pancreatic duct was obviously dilated, there were several slightly enlarged lymph nodes in the retroperitoneum, and metastasis was possible (Fig. 1). Since the onset of the disease, the patient had poor appetite and was in good general condition.

**Figure 1.** Enhanced CT before treatment: (A) a patchy slightly hypodense shadow was seen in the head and neck of the pancreas, with unclear borders and an extent of about 27 × 20 mm, with caudal atrophy of the body of the pancreas, marked dilatation of the corresponding pancreatic ducts, and no peripancreatic oozing was seen; (B) the proximal segment of the hepatic artery was encircled; (C) the abdominal trunk was encircled; (D) the portal vein was flattened by the compression, and the lumen did not have any obvious filling defects. CT = computed tomography.

The patient had undergone a partial left nephrectomy 10 years ago for a “left renal malformation tumor” and had no other previous medical history.

Preliminary diagnosis: pancreatic cancer with invasion of the PV, celiac trunk, and its branches; type II diabetes mellitus.

## 3. Therapeutic procedure

### 3.1. Neoadjuvant chemotherapy and percutaneous hepatic innominate artery embolization

Neoadjuvant chemotherapy with albumin-bound paclitaxel (200 mg + gemcitabine 1.4 g), injections on days 1 and 8, repeated every 3 weeks (albumin-paclitaxel + gemcitabine), was started in February 2023. Two months later, serum CA199 10.1 U/mL was reviewed (Fig. 2), and CT angiography of the mesenteric artery showed that the posterior peritoneal lymph nodes were slightly reduced compared to the previous one.

**Figure 2.** Trends in CA19-9 (yellow arrows: date of percutaneous hepatic innominate artery embolization; blue arrows: date of surgery).

After 3 cycles of neoadjuvant chemotherapy, the patient was evaluated for indications of surgical treatment, and the patient’s post-chemotherapy laboratory indicators were monitored until the liver function reached the standard. Percutaneous hepatic innominate artery embolization was performed on April 21, 2023 (see Fig. 3). There was no significant change in liver function after embolization compared with that before embolization. The 4th cycle of neoadjuvant chemotherapy was completed 13 days after embolization (Table 1). One month later, a follow-up enhanced CT scan of the upper abdomen showed a good hepatic blood supply, and collateral circulation of the perihepatic artery was successfully established (see Fig. 4).

**Table 1:** Four cycles of chemotherapy.

Chemotherapy cycle	1	2	3	4
Time	March 1, 2023	March 23, 2023	April 13, 2023	May 4, 2023

**Figure 3.** (A, B) Embolization of the hepatic innominate artery.

**Figure 4.** Enhanced CT – 1 mo after embolization: intrahepatic arterial blood flow is homogeneous throughout the liver.

### 3.2. Surgical process

Thirty-eight days after embolization, preoperative evaluation and preparation were improved, and total PD  + resection of the celiac trunk, common hepatic artery (CHA), and common hepatic innominate artery + PV resection and reconstruction + total gastrectomy + splenectomy + cholecystectomy + intestinal adhesion release were performed on May 29, 2023 (Fig. 5 for the surgical trauma). Among them are PV resection and reconstruction, celiac axis (CA) resection without reconstruction, and enlarged lymph node dissection. Intraoperatively, the splenic artery and the left gastric artery were blocked, and splenic and gastric ischemia were observed. The tissues around the CA and CHA and the root of the splenic artery became very stiff by invasion before chemotherapy, and the CA root was still available. Therefore, the CA transected at its root. The right and left hepatic arteries were ligated and dissected. The bile duct was then transected below the bifurcation. The PV, superior mesenteric vein (SMV), and splenic vein (2 cm in length) were resected and end-to-end anastomosis of the PV and SMV was performed. When dealing with the PV, due to tumor invasion, the vessel wall becomes fragile and heavily adherent to the surrounding tissues, which makes the separation and anastomosis of the vessel extraordinarily difficult. In order to ensure the smoothness of the anastomosis and the integrity of the vessels, fine microsurgical techniques were used to suture them layer by layer. Due to the enlargement and adhesion of the lymph nodes around the tumor, it was difficult to completely remove all the potentially involved lymph nodes by the traditional clearance method. Therefore, the strategy of extended lymph node dissection was used. Although this increases the complexity of the procedure, it can effectively reduce the risk of postoperative recurrence.

**Figure 5.** Surgical trauma (A) portal vein; (B) severed end of celiac axis; (C) inferior vena cava; and (D) abdominal aorta.

At this point, it was found that the tail of the pancreatic body, spleen, and gastric blood supply showed no signs of recovery; therefore, the tail of the pancreatic body, spleen, and remnants of the stomach were resected. Reconstruction of the digestive tract after total gastrectomy requires consideration of ways to minimize complications and restore the patient’s digestive function. We chose to perform an end-to-side anastomosis of the jejunum to the esophagus with a Brown anastomosis. Finally, a jejunostomy was performed. At the end of the operation, intraoperative Doppler ultrasound showed good arterial and portal venous blood flow to the entire liver. The procedure was uneventful, with an operative time of 535 minutes, intraoperative bleeding of approximately 800 mL, intraoperative transfusion of 2u of suspended red blood cells, and 320 mL of frozen plasma.

## 4. Postoperative condition

Enteral nutrition was started on the 3rd postoperative day, and the CT angiography of the mesenteric artery was reviewed on the 8th postoperative day. The wall of the abdominal aorta and its main branches of the CA, superior mesenteric artery, and bilateral renal arteries were smooth, with no stenosis or dilatation, and no signs of space occupation were observed. Postoperative pathological findings suggested middle and low differentiated ductal adenocarcinoma of the pancreatic head, the size of the tumor was 5 × 3 × 3 cm, infiltrating the pancreas and surrounding fibro-fatty tissues, and multifocal nerve invasion was observed locally. The margins of the incision were all negative, and no metastasis of the cancer was observed in the lymph nodes (0/7; metastasis/total number of lymph nodes). No tumors were observed in the gallbladder, spleen, duodenum, or stomach.

The patient started to show elevated alanine aminotransferase and menthyl aminotransferase on the 1st postoperative day, and after symptomatic treatment such as hepatoprotection was administered, they started to decrease gradually on the 2nd postoperative day. Fresh frozen plasma was transfused for 7 consecutive days after surgery to supplement coagulation factors (500 mL quaque die), and human albumin was transfused for 10 consecutive days (20 g quaque die; changes in postoperative laboratory indices are shown in Figs. 6–8). The patient was discharged from the hospital 20 days after surgery. The patient received oral pancreatic enzyme preparations and subcutaneous insulin regularly after the operation, with no occurrence of intractable diarrhea and stable blood glucose control. The patient has had tumor-free postoperative survival for more than 10 months, and her quality of life is acceptable.

**Figure 6.** Postoperative changes in AST and ALT. ALT = alanine aminotransferase, AST = aspartate aminotransferase.

**Figure 7.** Postoperative changes in total bilirubin, direct bilirubin, and indirect bilirubin.

**Figure 8.** Postoperative changes in prothrombinogen.

## 5. Discussion

It is publicly known that pancreatic cancer is one of the most malignant malignancies with the worst prognosis. Surgical resection is the only treatment for pancreatic cancer.^[4]^ The pancreas is anatomically deep and adjacent to large blood vessels in the upper abdomen. Pancreatic cancer progresses rapidly and the early symptoms are not typical; therefore, when the diagnosis is made, the blood vessels are often already invaded, and the chance of radical treatment is lost.

R0 resection is the most important criterion for ensuring the success of radical surgery for pancreatic cancer, and Ghaneh et al^[5]^ emphasized that R1 resection (positive margins) is independently associated with a reduction in overall survival (OS) and recurrence-free survival. Several studies have confirmed that R0 resection prolongs disease-free survival andOS.^[6,7]^

Vascular resection is an important step in achieving R0 resection in locally advanced pancreatic cancer with vascular invasion. In recent years, radical pancreatic cancer surgery combined with PV/SMV resection has been gradually performed in clinical practice, leading to a significant improvement in the survival of patients with locally advanced pancreatic cancer. Thus, is it possible to benefit patients with arterial involvement by combining arterial resection with radical pancreatic cancer surgery? Therefore, many surgeons and scholars at home and abroad have studied and explored this issue. Distal pancreatectomy with combined abdominal arterial resection (modified Appleby procedure) reported by several centers showed that combined arterial resection achieved a higher R0 resection rate, which can significantly prolong survival,^[8-10]^ and bring more benefits to patients with locally progressive pancreatic cancer relative to standard radical pancreatic cancer surgery. In 2017, a case of PD with combined hepatic arterial resection was reported by the Japanese scholar Miyazaki M.^[11]^ In 2022, Liang et al published the results of a study on autologous small-bowel transplantation for patients with superior mesenteric artery invasion. All these studies showed that radical pancreatic cancer surgery with combined arterial resection is safe and feasible in selected cases with adequate preoperative preparation and can improve the quality of life and long-term survival of patients.^[12]^

With the development of neoadjuvant chemotherapy in recent years, it brings more possibilities for radical resection of pancreatic cancer, Windsor JA et al^[13]^ showed that neoadjuvant chemotherapy may achieve tumor downstaging and increase the chances of R0 resection; Yoshiya S et al^[14]^ reported that the R0 resection rate could reach 81.8% after neoadjuvant chemotherapy. Xue et al reviewed 215 pancreatectomies (combined/non-combined preoperative neoadjuvant chemotherapy and arterial resection) and performed Mate analysis of their prognosis, which suggested that neoadjuvant chemotherapy followed by pancreatectomy with major arterial resection may improve survival in patients with unresectable pancreatic cancers involving arteries by achieving an R0 resection.^[15]^ A study carried out by Liang et al suggested that radical resection after NAT, combination of AR and small bowel transplantation produced a high R0 rate of 94.4% and an OS duration of 21.4 months.^[16]^

In this case, the PV, CA, and its branches were invaded by the tumor. After 4 cycles of neoadjuvant chemotherapy with the albumin-paclitaxel + gemcitabine, CA199 levels decreased by more than 50% of the initial value. Considering that the patient was effective on chemotherapy, the evaluation was followed by a planned surgical treatment. In this case, the PD combined with total abdominal trunk arterial resection was a long procedure, and the high level of difficulty and complexity of the procedure posed many technical challenges to the surgical team. First of all the vascularization was a critical part of the whole surgery. This case was preempted by percutaneous hepatic innominate artery embolization after evaluation, and the periportal hepatic arterial collateral circulation was established, which greatly reduced the possibility of severe hepatic failure due to hepatic ischemia in the postoperative period, while avoiding the need for hepatic artery reconstruction and simplifying the surgical procedure.^[11]^

A high rate of perioperative complications is a major concern in pancreatic cancer surgery. For radical pancreatic cancer surgery with combined arterial resection, the important factors determining its success are the patency of the arterial circulation and the presence of obstacles in the blood supply to the remaining abdominal organs. The 3 major branches of the CA are the splenic, left gastric, and common hepatic arteries. In this case, because of the intraoperative need to ligate the infringed celiac trunk and to dissociate the left gastric and splenic arteries, and because of the poor blood supply to the tail of the pancreatic corpuscle, spleen, and stomach, as revealed by the awaited assessment, the tail of the pancreatic corpuscle + the whole stomach + the spleen was resected to avoid delayed organ infarcts, infections, or abscesses.

In recent years, with the development and progress of surgical technology, dozens or even hundreds of ways have been developed to anastomose the digestive tract after pancreatectomy. In this case, after total gastrectomy, end-to-side anastomosis of jejunum and esophagus was performed by freeing and lifting up jejunum, and Brown anastomosis was performed by input loop and output loop, which could reduce bile reflux and anastomotic ulcer.^[17]^ This type of reconstruction is complex, but tacit teamwork and intraoperative skillful operation can effectively shorten the operation time and improve the patients’ postoperative quality of life.

Internal and external secretory insufficiency after total PD remains a difficult problem; however, due to technological advances, postoperative glycemia can be better controlled. In this case, long-acting insulin and short-acting insulin were used in combination after surgery, and blood glucose control has been stable since the follow-up, which did not have a significant impact on the quality of life after surgery. Diarrhea is the most common complication after total pancreatectomy; however, with the postoperative adjustment of the patient’s dietary habits, improvement of nutritional status, and optimization of pancreatic enzyme therapy, most patients will not develop persistent diarrhea. This patient had frequent but mostly formed stools, and no significant weight loss was observed. Overall, the impact of post-total pancreatectomy complications on postoperative quality of life was within acceptable limits.

In conclusion, the development of new concepts in drugs, imaging, pathology, and surgery for pancreatic cancer has provided new opportunities and advances in the treatment of pancreatic cancer. In cases of pancreatic cancer invading the abdominal trunk and CHA, radical resection of pancreatic cancer combined with vein resection under adequate preoperative preparation has shown good recent results. However, the available research data are still limited; therefore, further studies need to be performed in a standardized manner in more experienced large pancreatic centers to confirm this idea.

## Author contributions

**Conceptualization:** Bin Zhang, Ying’an Zhao, Xuanlei Ren, Siming Zheng.

**Data curation:** Mengna Zhang, Bin Zhang, Ying’an Zhao, Jiyun Zhu, Xuanlei Ren, Jianbo Zheng.

**Formal analysis:** Mengna Zhang, Jiyun Zhu, Jianbo Zheng.

**Investigation:** Xuanlei Ren, Jianbo Zheng.

**Methodology:** Bin Zhang, Ying’an Zhao, Anle Wu.

**Project administration:** Siming Zheng.

**Software:** Mengna Zhang.

**Supervision:** Ying’an Zhao, Anle Wu, Jiyun Zhu, Siming Zheng.

**Validation:** Siming Zheng.

**Writing – original draft:** Mengna Zhang.

**Writing – review & editing:** Siming Zheng.
